The article "Protective Role of Taurine against Arsenic-Induced Mitochondria-Dependent Hepatic Apoptosis via the Inhibition of PKCδ-JNK Pathway" was retracted in 2025. Reasons: errors in the images; duplicated images; overlap with earlier publications; original data or images not available.

# Protective Role of Taurine against Arsenic-Induced Mitochondria-Dependent Hepatic Apoptosis via the Inhibition of PKCδ-JNK Pathway

**DOI:** 10.1371/journal.pone.0012602

**Published:** 2010-09-07

**Authors:** Joydeep Das, Jyotirmoy Ghosh, Prasenjit Manna, Parames C. Sil

**Affiliations:** Division of Molecular Medicine, Bose Institute, Kolkata, India; Technical University Munich, Germany

## Abstract

**Background:**

Oxidative stress-mediated hepatotoxic effect of arsenic (As) is mainly due to the depletion of glutathione (GSH) in liver. Taurine, on the other hand, enhances intracellular production of GSH. Little is known about the mechanism of the beneficial role of taurine in As-induced hepatic pathophysiology. Therefore, in the present study we investigated its beneficial role in As-induced hepatic cell death via mitochondria-mediated pathway.

**Methodology/Principal Findings:**

Rats were exposed to NaAsO_2_ (2 mg/kg body weight for 6 months) and the hepatic tissue was used for oxidative stress measurements. In addition, the pathophysiologic effect of NaAsO_2_ (10 µM) on hepatocytes was evaluated by determining cell viability, mitochondrial membrane potential and ROS generation. As caused mitochondrial injury by increased oxidative stress and reciprocal regulation of Bcl-2, Bcl-xL/Bad, Bax, Bim in association with increased level of Apaf-1, activation of caspase 9/3, cleavage of PARP protein and ultimately led to apoptotic cell death. In addition, As markedly increased JNK and p38 phosphorylation with minimal disturbance of ERK. Pre-exposure of hepatocytes to a JNK inhibitor SP600125 prevented As-induced caspase-3 activation, ROS production and loss in cell viability. Pre-exposure of hepatocytes to a p38 inhibitor SB2035, on the other hand, had practically no effect on these events. Besides, As activated PKCδ and pre-treatment of hepatocytes with its inhibitor, rottlerin, suppressed the activation of JNK indicating that PKCδ is involved in As-induced JNK activation and mitochondrial dependent apoptosis. Oral administration of taurine (50 mg/kg body weight for 2 weeks) both pre and post to NaAsO_2_ exposure or incubation of the hepatocytes with taurine (25 mM) were found to be effective in counteracting As-induced oxidative stress and apoptosis.

**Conclusions/Significance:**

Results indicate that taurine treatment improved As-induced hepatic damages by inhibiting PKCδ-JNK signalling pathways. Therefore taurine supplementation could provide a new approach for the reduction of hepatic complication due to arsenic poisoning.

## Introduction

Arsenic (As) is a widespread environmental toxin. It enters the organisms by dermal contact, inhalation, or ingestion of contaminated drinking water and affects nearly entire organ systems of the body [1]. Investigations at the cellular and molecular levels reveal that As enhances production of reactive oxygen species (like, superoxide and hydrogen peroxide), causes lipid peroxidation, enhances oxidation of proteins, enzymes as well as DNA [2], [3], disrupts mitosis and promotes apoptosis [4]. Among several mechanisms, oxidative stress due to accelerated production of free radicals has also been implicated for As-induced injury in liver, kidney, brain, testes and other tissues [5], [6].

The article "Protective Role of Taurine against Arsenic-Induced Mitochondria-Dependent Hepatic Apoptosis via the Inhibition of PKCδ-JNK Pathway" was retracted in 2025. Reasons: errors in the images; duplicated images; overlap with earlier publications; original data or images not available.

Antioxidants have been found beneficial to mitigate chemical-induced oxidative damage [7], [8], [9], [10]. Antioxidant property of the conditional amino acid, taurine (2-aminoethanesulfonic acid), is also well-established and therefore, could be considered as a potent candidate in this regard. Taurine is an end product of L-cysteine metabolism and is the most abundant free amino acid in many tissues. It protects many of the body's organs against toxicity and oxidative stress caused by various toxic substances [11], [12], [13], [14], [15], [16], [17]. Taurine causes enhancement in intracellular glutathione (GSH) levels by directing cysteine into the GSH synthesis pathways as cysteine is a precursor of both taurine and GSH [18], [19]. Taurine also stabilizes GSH-metabolizing enzymes [20], stimulates glucose-6-phosphate dehydrogenase that generates NADPH needed for the restoration of GSH from GSSG [21]. Since the hepatotoxic effect of As is mainly due to the depletion of GSH in the liver, hence, it may be hypothesized that taurine could also play a protective role against As-induced hepatotoxicity.

The drinking water containing arsenic more than 10 µg/L is harmful to the body. In human, signs of chronic toxicity appear after long term exposure to a low dose of arsenic and thus we selected comparatively higher dose of arsenic in the present study using a rat model for achieving similar effects seen in humans. Therefore, the chronic arsenic toxicity in rats was achieved by oral administration of NaAsO_2_ at a dose of 2 mg/kg body weight, approximately 25 ppm in distilled water for 6 months [22]. The present study has been undertaken to evaluate the beneficial role of taurine in As-induced hepatic pathophysiology using both in vivo and in vitro models by measuring in vivo antioxidant power, levels of cellular metabolites (GSH, GSSG), activities of antioxidant enzymes, lipid peroxidation end products etc. Molecular mechanism underlying the protective action of taurine against NaAsO_2_ induced hepatic dysfunction was assessed by evaluating the role of different PKC isoforms and MAP kinase family proteins. In addition, anti-apoptotic action of taurine was evaluated by measuring the mitochondrial membrane potential, intracellular ATP level, DNA fragmentation, alterations of the Bcl-2 family proteins, Bim, cytosolic cytochrome C, activities of Apaf-1, caspase 9, caspase 3, and PARP. The results of the present study could clarify the role of this important bioactive molecule in the prevention of As-induced hepatotoxicity, and may shed light on a possible solution to the serious hepatic complications arising due to As exposure.

The article "Protective Role of Taurine against Arsenic-Induced Mitochondria-Dependent Hepatic Apoptosis via the Inhibition of PKCδ-JNK Pathway" was retracted in 2025. Reasons: errors in the images; duplicated images; overlap with earlier publications; original data or images not available.

## Results

### Dose dependent effect of NaAsO_2_ by ALP assay

In order to determine the dose-dependent As induced hepatic damage, we carried out a dose-dependent study using ALP assay as an index of that damage. As evidenced from figure 1A, in As intoxicated animals, maximum ALP level in plasma was reached at a dose of 2 mg/kg body weight after 6 months. Effect of As was not much beyond this concentration. This dose was, therefore, chosen as for As-induced hepatic damage throughout the study.

**Figure 1:** Dose and time dependant effect of NaAsO_2_ and taurine. Panel A: Dose dependant effect of NaAsO_2_ on ALP level. Cont: ALP level in normal rats; As-0.5, As-1, As-1.5, As-2, As-2.5, As-3: ALP level in NaAsO_2_ intoxicated rats at a dose of 0.5 mg, 1 mg, 1.5 mg, 2 mg, 2.5 mg and 3 mg/kg body weight respectively for 6 months. Panel B: Dose and time dependent effect of taurine on ALP level against arsenic induced toxicity. Cont: ALP level in normal rats, As: ALP level in NaAsO_2_ treated rats, TAU-10+As, TAU-20+As, TAU-30+As, TAU-40+As, TAU-50+As, TAU-60+As: ALP level in taurine (TAU) treated rats for 2 weeks at a dose of 10, 20, 30, 40, 50 and 60 mg/kg body weight prior to NaAsO_2_ administration; TAU-0.5W+As, TAU-1W+As, TAU-1.5W+As, TAU-2W+As, TAU-2.5W+As, TAU-3W+As: ALP level in taurine (TAU) treated rats for 0.5, 1, 1.5, 2, 2.5 and 3 weeks respectively at a dose of 50 mg/kg body weight prior to As administration. Panel C: Time dependent effect of taurine on ALP level against NaAsO_2_ induced toxicity in serum. Cont: ALP level in normal rats, As-0.5W, As-1W, As-2W, As-2.5W, As-3W: ALP level in NaAsO_2_ intoxicated rats after 0.5, 1, 2, 2.5 and 3 weeks respectively from the last dose of NaAsO_2_, As+TAU-0.5W, As+TAU-1W, As+TAU-1.5W, As+TAU-2.5W, As+TAU-3W: ALP level in taurine (TAU) treated rats for 0.5, 1, 2, 2.5 and 3 weeks respectively at a dose of 50 mg/kg body weight after NaAsO_2_ administration. Each column represents mean ± SD, n = 6. “a” indicates the significant difference between the normal control and As intoxicated groups and “b” indicates the significant difference between taurine post-treated and recovery groups. (P^a^<0.05, P^b^<0.05).

The article "Protective Role of Taurine against Arsenic-Induced Mitochondria-Dependent Hepatic Apoptosis via the Inhibition of PKCδ-JNK Pathway" was retracted in 2025. Reasons: errors in the images; duplicated images; overlap with earlier publications; original data or images not available.

### Dose and time dependent study of taurine by ALP assay

ALP assay was used to determine the optimum dose and time necessary for taurine to protect rat liver against NaAsO_2_ induced oxidative damages. Experimental results suggest that NaAsO_2_ intoxication (at a dose of 2 mg/kg body weight for, orally for 6 months) increased the ALP level and that could be prevented by the pretreatment with taurine up to a dose of 50 mg/kg body weight daily for 2 weeks (figure 1B).

Similarly post-treatment with taurine at a dose of 50 mg/kg body weight daily for 2 weeks after NaAsO_2_ administration also decreased the elevated level of ALP (figure 1C). These dose and time were, therefore, chosen as the optimum dose and time for taurine treatment throughout the study.

### Effect of taurine on As-induced hepatotoxicity

To elucidate whether NaAsO_2_ administration induced liver damage, we measured food intake, body weight, liver weight and the serum specific marker enzymes activities. During the 6 months of exposure of arsenic, no mortality occurred. There was no significant difference in food and water intake between normal and NaAsO_2_ exposed animals. Body weight and liver weight were reduced in NaAsO_2_ exposed animals compared to control animals although the liver weight to body weight ratios between these two groups remained practically unaltered (table 1). Both Pre and post-treatment with taurine significantly inhibited this alteration of the liver and body weight.

**Table 1:** Effect of taurine on NaAsO_2_- induced hepatotoxicity in experimental rats.

Parameters	Normal Control	Toxin Control	TAU+As	As+TAU	TAU
Body weight(g)	265.25±6.27	237.72±5.16^a^	259.78±5.98^b^	252.59±5.77^b^	267.54±6.27
Liver weight(g)	5.71±0.16	5.12±0.13	5.48±0.14	5.40±0.14	5.72±0.17
Ratio of the liverWeight to the body weight (%)	2.16±0.13	2.15±0.13	2.11±0.14	2.14±0.14	2.14±0.14
Hepatic Arsenic (µg/g tissue)	0.16±0.01	1.54±0.06^a^	0.52±0.03^b^	0.69±0.03^b^	0.13±0.01
Urinary Arsenic (µg/g creatinine)	7.86±0.31	61.13±2.57^a^	118.47±4.92^b^	103.37±4.09^b^	10.51±0.48
ALT (IU/L)	20.54±0.06	38.52±1.53^a^	24.24±1.12^b^	26.75±1.27^b^	20.15±0.08
ALP (KA Units)	27.58±1.23	55.26±3.21^a^	32.39±2.03^b^	36.38±2.05^b^	25.49±0.83

“a” values differs significantly from normal control (P^a^<0.05).

“b” values differs significantly from toxin control (P^b^<0.05).

Values are expressed as mean ± SD, for 6 animals in each group.

We observed increased deposition of arsenic in the liver of arsenic exposed animals, thus indicating the incapability of the liver to eliminate the increased arsenic that the animals were exposed to (table 1). Taurine effectively increased urinary arsenic excretion and thus lowered the accumulation of arsenic in the liver tissues (table 1). The status of the serum specific marker enzymes related to liver dysfunctions has been represented in table 2. NaAsO_2_ administration caused a significant increase in the activities of ALT and ALP (table 1). However, taurine treatment both pre and post to NaAsO_2_ administration reduced these levels almost close to normal against NaAsO_2_ induced hepato-toxicity.

The article "Protective Role of Taurine against Arsenic-Induced Mitochondria-Dependent Hepatic Apoptosis via the Inhibition of PKCδ-JNK Pathway" was retracted in 2025. Reasons: errors in the images; duplicated images; overlap with earlier publications; original data or images not available.

**Table 2:** Effect of taurine on NaAsO_2_-induced mitochondrial oxidative stress.

Parameters	Normal Control	Toxin Control	TAU+As	As+TAU	TAU
GSH (nmol/mg protein)	8.32±0.37	4.82±0.27^a^	7.86±0.33^b^	6.41±0.28^b^	9.18±0.41
GSSG (nmol/mg protein)	0.19±0.01	0.54±0.03^a^	0.23±0.01^b^	0.28±0.01^b^	0.17±0.008
Redox ratio (GSH/GSSG)	43.79±2.12	8.92±0.52^a^	34.17±1.63^b^	22.89±1.11^b^	54.0±2.31
MDA (nmol/mg protein)	3.79±0.15	7.53±0.34^a^	4.62±0.21^b^	5.14±0.22^b^	3.15±0.14

“a” values differs significantly from normal control (P^a^<0.05).

“b” values differs significantly from toxin control (P^b^<0.05).

Values are expressed as mean ± SD, for 6 animals in each group.

### As-induced hepatic oxidative stress: protection by taurine

GSH plays a critical role in scavenging ROS generated after the toxic insult. A massive amount of GSH is consumed to accomplish this task, thus shifting the redox status of the cell. Similar results were exhibited in our study in which NaAsO_2_ drastically reduced GSH/GSSG ratio by 4.9-fold (table 2) in liver mitochondria and 5.3-folds (table 3) in liver tissue confirming ROS generation and oxidative stress. In addition we also found that peroxidation of both mitochondrial (table 2) and total cellular lipid (table 3) increased significantly in the liver following NaAsO_2_ administration. Treatment with taurine, however, maintained these levels almost close to normal. Our results also indicated that administration of taurine increases activities of antioxidant enzymes (catalase, GST, GPx, GR, SOD and G6PD) compared to NaAsO_2_ exposed animals (table 4). Increase in the activities of these enzymes prevents the mitochondrial generated reactive radicals from causing oxidative stress, cellular damage and compensate for lack of GSH functioning.

**Table 3:** Effect of taurine on NaAsO_2_-induced oxidative stress in liver tissue.

Parameters	Normal Control	Toxin Control	TAU+As	As+TAU	TAU
GSH (nmol/mg protein)	17.36±0.826	8.51±0.38^a^	15.69±0.71^b^	13.19±0.55^b^	18.58±0.82
GSSG (nmol/mg protein)	0.34±0.02	0.89±0.04^a^	0.41±0.02^b^	0.47±0.02^b^	0.31±0.01
Redox ratio (GSH/GSSG)	51.06±2.23	9.56±0.42^a^	38.27±1.85^b^	28.06±1.19^b^	59.94±2.29
MDA (nmol/mg protein)	3.25±0.13	6.51±0.31^a^	4.01±0.20^b^	4.24±0.19^b^	3.07±0.12
H_2_O_2_ (nmol/mg liver)	1.46±0.06	3.16±0.09^a^	1.83±0.08^b^	1.99±0.04^b^	1.32±0.07

“a” values differs significantly from normal control (P^a^<0.05).

“b” values differs significantly from toxin control (P^b^<0.05).

The article "Protective Role of Taurine against Arsenic-Induced Mitochondria-Dependent Hepatic Apoptosis via the Inhibition of PKCδ-JNK Pathway" was retracted in 2025. Reasons: errors in the images; duplicated images; overlap with earlier publications; original data or images not available.

Values are expressed as mean ± SD, for 6 animals in each group.

**Table 4:** Effect of taurine and NaAsO_2_ on the activities of the antioxidant enzymes.

Name of the antioxidant enzymes	Activities of the antioxidant enzymes				
	Normal Control	Toxin Control	TAU+As	As+TAU	TAU
SOD (Unit/mg protein)	116.42±5.13	63.57±3.02^a^	106.97±4.82^b^	91.76±4.21^b^	121.18±5.14
CAT (µmol/min/mg protein)	189.22±8.63	89.78±3.52^a^	167.96±7.52^b^	159.76±6.83^b^	192.48±8.71
GST (µmol/min/mgprotein)	3.59±0.15	1.16±0.05^a^	2.34±0.12^b^	2.12±0.10^b^	3.67±0.16
GR (nmol/min/mgprotein)	144.91±6.82	66.36±3.23^a^	119.94±5.21^b^	109.48±4.93^b^	146.42±6.83
GPx. (nmol/min/mgprotein)	157.05±7.32	69.91±3.21^a^	144.51±6.82^b^	137.41±6.57^b^	159.43±7.31
G6PD (nmol/min/mgprotein)	241.69±10.29	132.51±6.39^a^	223.62±9.68^b^	217.05±9.18^b^	246.18±10.30

“b” values differs significantly from normal control (P^a^<0.05).

“b” values differs significantly from toxin control (P^b^<0.05).

Values are expressed as mean ± SD, for 6 animals in each group.

### Effects of taurine against NaAsO_2_-induced H_2_O_2_ level

Arsenic-induced oxidative stress has been shown to cause DNA damage through the production of superoxide and hydrogen peroxide. Therefore, we measured the H_2_O_2_ level in hepatic tissues of the experimental animals. We observed that hepatic H_2_O_2_ level was significantly increased in NaAsO_2_ exposed animals (table 4). However, treatment with taurine both pre and post to NaAsO_2_ administration reduced this H_2_O_2_ production.

### Taurine ameliorated As induced cytotoxicity

Our results showed that NaAsO_2_ caused loss in cell (hepatocytes) viability. To investigate whether this loss could be prevented by taurine, we performed MTT assay. As evidenced from figure 2A, reduction in cell viability increased with increasing NaAsO_2_ concentration. Incubation of the hepatocytes with NaAsO_2_ at a concentration of 10 µM for 8 hr showed optimum reduction in cell viability. After that, the loss in cell viability remains practically constant even with increasing NaAsO_2_ concentration. Therefore, this particular concentration of NaAsO_2_ has been used throughout the study. Figure 2B showed that the increased taurine concentration (from 5 to 30 mM), caused a dose dependent increase in viability of NaAsO_2_ treated cells. While NaAsO_2_ exposed hepatocytes had a viability of only 62%, taurine treatment increased the viability upto 93% when treated with 25 mM (optimum concentration) taurine. Therefore, this concentration (25 mM) of taurine has been used in all the subsequent studies.

The article "Protective Role of Taurine against Arsenic-Induced Mitochondria-Dependent Hepatic Apoptosis via the Inhibition of PKCδ-JNK Pathway" was retracted in 2025. Reasons: errors in the images; duplicated images; overlap with earlier publications; original data or images not available.

**Figure 2:** Impact of As and taurine on cell viability, ROS production, Δψ_m_ and intracellular ATP levels. Panel A: Dose dependent effect of As on cell viability; Panel B: Dose dependent effect of taurine on As treated hepatocytes; Cont: cell viability in normal hepacytes; As-2.5, As-5, As-7.5, As-10, As-12.5 and As-15: cell viability in As treated hepatocytes for 8 h at a dose of 2.5, 5, 7.5, 10, 12.5 and 15 µM; TAU-10, TAU-20, TAU-25, TAU-30, and TAU-40: cell viability level in hepatocytes treated with taurine (1 h prior to As addition) and As for 8 h at a dose of 10, 20, 25, 30 and 40 mM. Panel C: The intracellular ROS production was detected by DCF-DA method in As treated hepatocytes in absence (As) and presence of taurine (TAU+As). SP600125+As: ROS production in hepatocytes treated with 10 µM SP600125 15 minutes before As exposure and incubated for 8 h, SP600125+TAU+As: ROS production in hepatocytes treated with 10 µM SP600125 and 25 mM taurine 15 minutes before As exposure and incubated for 8 h. Arrows indicate fluorescent dye, DCF uptake by hepatocytes. We have taken equal number of cells in each set as observed in microscope under bright field. Panel D: mitochondrial membrane potential (Δψ_m_) was measured using a fluorescent cationic probe rhodamine-123 by flow cytometer with FL-1 filter. Results represent one of the six independent experiments. Panel E: Effect of taurine on As-induced decrease in intracellular ATP levels. CON, ATP levels in untreated hepatocytes; As: ATP levels in hepatocytes treated with As; TAU+As: ATP levels in hepatocytes treated with taurine along with As. “a” indicates the significant difference between the normal control and toxin-treated cells, “b” indicates the significant difference between toxin control and taurine-treated cells. Each column represents mean ±SD, n = 6; (p^a^<0.05, p^b^<0.05).

Earlier experiments suggest that NaAsO_2_ induces reactive oxygen species (ROS) generation in the liver tissue of experimental animals [23]. So, we wanted to find out whether this toxin could exert the same effect in the liver cells, hepatocytes and if it could, whether taurine plays any protective role in this pathophysiology. We, therefore, determined the ROS level in all sets of experimental hepatocytes (normal, As-treated and taurine+As treated). Fluorescence spectrometric analysis showed that NaAsO_2_ enhanced ROS generation in hepatocytes (Fig. 2C), (arrows indicate fluorescent dye, DCF uptake by hepatocytes) and that could be prevented by treatment with taurine.

The article "Protective Role of Taurine against Arsenic-Induced Mitochondria-Dependent Hepatic Apoptosis via the Inhibition of PKCδ-JNK Pathway" was retracted in 2025. Reasons: errors in the images; duplicated images; overlap with earlier publications; original data or images not available.

Mitochondrial membrane potential (Δψ_m_) was assessed in the liver mitochondria of NaAsO_2_ exposed hepatocytes. Δψ_m_ was decreased in mitochondria isolated from the hepatocytes exposed with As (Fig. 2D). Administration of taurine prevented this NaAsO_2_-induced loss in Δψ_m_ thereby indicating the membrane stabilizing effect of taurine.

In addition, cellular ATP level was also measured and found that this level was significantly lower in As-exposed hepatocytes than in untreated ones (Fig. 2E). However, pretreatment of hepatocytes with taurine could prevent this As-induced lowering of ATP content.

Loss of the mitochondrial membrane potential promotes cytochrome c release into cytosol and activates caspases via apoptosome formation. Therefore, we assessed the leakage of cytochrome c into cytosol and the status of caspases (initiator caspase 9 and effector caspase 3) and Apaf-1 in NaAsO_2_ intoxicated hepatocytes. Immunoblot analyses showed an decreased mitochondrial cytochrome c level, increased cytosolic cytochrome c and Apaf-1 level associated with up-regulation of caspase 9, caspase 3 and cleaved caspase 3 in NaAsO_2_ exposed hepatocytes indicating involvement of the mitochondrial apoptotic pathway in this pathophysiology (figure 3A, 3B, 3C, 3D, 3E). Taurine exerted its beneficial effect by inhibiting cytochrome c release and Apaf-1. It was also found to be effective in inhibiting caspase 3 and caspase 9 levels in the cytosol.

**Figure 3:** Immunoblot analysis on Mitochondrion-dependent pathway in absence (As) and presence of taurine (TAU+As). Panel A: Mitochondrial cytochrome c, complex IV subunit was used as loading control. Panel B: Cytosolic cytochrome c, Panel C: Caspase 9, Panel D: Apaf 1, Panel E: Caspase 3, Panel F: PARP. β actin was used as an internal control. Data represent the average ± SD of 6 separate experiments in each group. “a” indicates the significant difference between the normal control and As treated groups, “b” indicates the significant difference between the As treated and taurine treated groups (TAU+As). (P^a^<0.05, P^b^<0.05).

We then examined PARP cleavage to elucidate the molecular mechanism underlying the protective effects of taurine against NaAsO_2_-induced cell death as PARP cleavage represents a biochemical hallmark of apoptosis. Western blot analysis revealed that NaAsO_2_ exposure caused the degradation of 116 kDa PARP to the characteristic 84 kDa PARP fragment (figure 3F). However, taurine treatment could inhibit this NaAsO_2_-induced cleavage of PARP.

### As-induced apoptosis of hepatocytes: modulation by taurine

We, further, investigated the mode of cell death in hepatocytes isolated from NaAsO_2_-exposed rats using flow cytometric analysis, DNA gel electrophoresis and DAPI staining. To characterize the nature of NaAsO_2_-induced cell death pathway, we, first quantified apoptotic cells among the injured ones using flow cytometry analysis. As illustrated in Figure 4A, about 55.23% of the hepatocytes isolated from NaAsO_2_-exposed rats underwent apoptosis, among which 38.74% hepatocytes underwent early apoptosis (annexin V^+^/PI^−^), 16.49% hepatocytes underwent late apoptosis (annexin V^+^/PI^+^) and 11.20% hepatocytes underwent necrosis (annexin V^−^/PI^+^). However both pre and post-treatment with taurine (hepatocytes viability are respectively 81.89% and 74.48%) effectively reduced the numbers of both apoptotic and necrotic cells indicating that taurine protected hepatocytes in NaAsO_2_-induced hepatic pathophysiology.

The article "Protective Role of Taurine against Arsenic-Induced Mitochondria-Dependent Hepatic Apoptosis via the Inhibition of PKCδ-JNK Pathway" was retracted in 2025. Reasons: errors in the images; duplicated images; overlap with earlier publications; original data or images not available.

**Figure 4:** Mode of cell death in absence (As) and presence of taurine (TAU+As and As+TAU). Fig. A: percent distribution of apoptotic and necrotic cells. Cell distribution was analysed using Annexin V binding (taken as x axis) and PI uptake (taken as y axis). The FITC and PI fluorescence were measured using flow cytometer with FL-1 and FL-2 filters respectively. Results expressed as dot plot representing as one of the six independent experiments. Fig. B: DNA fragmentation pattern on agarose/EtBr gel. DNA isolated from experimental liver tissues was loaded onto 1% (w/v) agarose gels. Lane 1: Marker (1 kb DNA ladder); Lane 2: DNA isolated from normal liver; Lane 3: DNA isolated from As intoxicated liver; Lane 4: DNA isolated from taurine pretreated liver samples, Lane 5: DNA isolated from taurine post-treated liver samples. Arrows indicate ladder formation in DNA isolated from NaAsO_2_ intoxicated animals. Fig. C: DAPI staining. Cell nuclei of untreated or As and taurine treated hepatocytes were visualized following DNA staining with the fluorescent dye DAPI and were observed using a microscope (original magnification ×20). The measurements were made in six times. Arrows indicate fragmented and condensed DNA in hepatocytes.

Next, to show the apoptotic changes in the hepatocytes, we examined the DNA fragmentation pattern. NaAsO_2_ caused a DNA ladder fragmentation (a hallmark of apoptosis) associated with a smear (figure 4B). Taurine treatment effectively reduced the DNA laddering and smearing of the NaAsO_2_ exposed animals.

Finally we focused on the morphological changes of hepatocytes undergoing apoptosis (induced by NaAsO_2_) using DAPI staining. As shown in Figure 4C, hepatocytes from control animals exhibit normal morphology, whereas cells from NaAsO_2_ exposed animals were observed to have condensed and fragmented DNA in the nucleus. Taurine treatment, however, restored the normal morphology of these cells as evidenced from the figure 4C.

The article "Protective Role of Taurine against Arsenic-Induced Mitochondria-Dependent Hepatic Apoptosis via the Inhibition of PKCδ-JNK Pathway" was retracted in 2025. Reasons: errors in the images; duplicated images; overlap with earlier publications; original data or images not available.

### Taurine mitigated the pro-apoptotic effects of As on Bcl-2 family and BH3-only proteins

Oxidative stress-induced apoptosis is directly related to mitochondrial dysfunction. Therefore, we investigated whether As-induced mitochondrial dysfunction is mediated by the Bcl-2 family proteins. We observed that NaAsO_2_ induced up-regulation of pro apoptotic (active non-phospho form of Bad, Bax) and down-regulation of anti apoptotic (active non-phospho form of Bcl-2, Bcl-xL) Bcl-2 family proteins both in vivo and in vitro (Fig. 5A, 5B, 5C, 5D). However, taurine treatment inhibited As-induced up-regulation of Bad, Bax and down-regulation of Bcl-2, Bcl-xL. To further investigate whether arsenic exposure affects the expression of Bcl-2 and Bax at the mRNA levels, transcription levels of Bcl-2 and Bax were checked in the liver tissue of the experimental rats. Semi-quantitative analysis showed significant down regulation of Bcl-2 gene and upregulation of Bax gene expressions following arsenic exposure. However, these altered gene expressions were reversed due to taurine treatment. Of the eight known BH3-only proteins, only Bim and Bid bind and activate Bax. Since in the present study, we set our aim to investigate mitochondrion dependent apoptotic pathways and “Bid” is not involved in this pathway, we investigated the effect of “arsenic and taurine” on “Bim” in hepatocytes apoptosis. Bim exists at the protein level as three isoforms, including Bim extra long (BimEL), Bim long (BimL), and Bim short (BimS). In the liver and hepatocytes, BimEL was readily identified by immunoblot analysis. Arsenic significantly increased cellular BimEL protein expression, whereas treatment with taurine could reduce this alteration (Fig. 5E).

**Figure 5:** Immunoblot analysis on Bcl-2 family and Bim in response to As and taurine (TAU+As, As+TAU). Panel A: Bax, Panel B: Bad, Panel C: Bcl-2, Panel D: Bcl-xL, Panel E: Bim-EL. β actin was used as an internal control. Panel F: Tissue expression of mRNAs for Bax and Bcl-2 in livers isolated from normal as well as NaAsO_2_ and taurine treated rats. β actin was taken as an internal control. Data represent the average ± SD of 6 separate experiments in each group. “a” indicates the significant difference between the normal control and As treated groups, “b” indicates the significant difference between the As treated and taurine treated groups. (P^a^<0.05, P^b^<0.05).

### Activation of MAP kinase by NaAsO_2_, protection via Taurine

To investigate whether MAPKs play any role in As-induced hepatic pathophysiology and apoptotic cell death, we first analyzed the activation status of ERK1/2, JNK, and p38 MAPK by immunoblot analyses with antibodies specific to the phosphorylated form of these kinases. NaAsO_2_ intoxication resulted in a dramatic increase in the phosphorylated form of p38 and JNK MAPKs in both rat liver and hepatocytes (Fig. 6). On the other hand, the level of the phosphorylated ERK1/2 was not altered significantly. However, taurine treatment both pre and post to NaAsO_2_ administration significantly reduced all these As induced alterations.

The article "Protective Role of Taurine against Arsenic-Induced Mitochondria-Dependent Hepatic Apoptosis via the Inhibition of PKCδ-JNK Pathway" was retracted in 2025. Reasons: errors in the images; duplicated images; overlap with earlier publications; original data or images not available.

**Figure 6:** Immunoblot analysis on MAPKinase family proteins in response to As and taurine (TAU+As and As+TAU). Panel A: Phospho and total JNK, Panel B: Phospho and total p38, Panel C: Phospho and total ERK1/2. β actin was used as an internal control. Data represent the average ± SD of 6 separate experiments in each group. “a” indicates the significant difference between the normal control and As treated groups, “b” indicates the significant difference between the As treated and taurine treated groups. (P^a^<0.05, P^b^<0.05).

### Effects of p38 and JNK MAPK inhibition on As-induced apoptosis

Based on the earlier result, we investigated whether p38 and JNK MAPKs are involved in the prevention of As-induced apoptosis in hepatocytes. The cells were pre-treated with SB203580, SP600125 separately for 15 min for two different sets of experiments and then effect of As on cell viability and caspase-3 activation were determined. Results showed that JNK inhibition significantly increased cell viability and reduced caspase-3 activation in NaAsO_2_ exposed hepatocytes, where as p38 inhibition had no effect on these events (Fig. 7), indicating that p38-MAPK is not involved in the prevention of As-induced apoptosis. In presence of the JNK inhibitior, NaAsO_2_ did not cause any significant change in ROS generation (Fig. 2C). When cells were treated with taurine in presence of JNK inhibitor, further reduction in ROS production (Fig. 2C) and caspase-3 inactivation were observed accompanied by an increase in cell viability (Fig. 7), suggesting the involvement of JNK MAPK signaling pathway in taurine mediated cyto protection.

**Figure 7:** Immunoblot analysis of caspase 3 and hepatocytes viability in response to SB203580 and SP600125. Hepatyocytes were pre-treated with 10 µM SB203580 and SP600125 for 15 min, then treated with As (10 µM), taurine (25 mM, added 1 h prior to As treatment) for 8 h. Panel A: effects of SP600125 on Caspase 3, Panel B: effects of SB203580 on Caspase 3, β actin was used as an internal control. Panel C: effects of SP600125 on cell viability, Panel D: effects of SB203580 on cell viability. Data represent the average ± SD of 6 separate experiments in each group. “a” indicates the significant difference between the normal control and As treated groups, “b” indicates the significant difference between the As treated and taurine treated groups. (P^a^<0.05, P^b^<0.05).

The article "Protective Role of Taurine against Arsenic-Induced Mitochondria-Dependent Hepatic Apoptosis via the Inhibition of PKCδ-JNK Pathway" was retracted in 2025. Reasons: errors in the images; duplicated images; overlap with earlier publications; original data or images not available.

### Activation of PKC by NaAsO_2_, inhibition by taurine

The PKC family consists of a number of different serine/threonine kinases, of which specific isoforms have been shown to be either pro-apoptotic or anti-apoptotic, depending on the nature of the stimuli and cell types used for the study [24], [25], [26], [27]. We, therefore, determined the role of major PKC isoforms in As induced hepatic pathophysiology and observed that NaAsO_2_ intoxication significantly increased the expression of PKCδ both in vivo and in vitro, where as the expression of other two major isoforms of PKC, (PKCα and PKCξ) remained unchanged (Fig. 8). Taurine treatment, however, significantly reduced this As induced up-regulation of PKCδ.

**Figure 8:** Immunoblot analysis of PKC family proteins in response to As and taurine (TAU+As and As+TAU). Panel A: Phospho and total PKCα, Panel B: Phospho and total PKCδ, Panel C: Phospho and total PKCξ. Data represent the average ± SD of 6 separate experiments in each group. β actin was used as an internal control. “a” indicates the significant difference between the normal control and As treated groups, “b” indicates the significant difference between the As treated and taurine treated groups. (P^a^<0.05, P^b^<0.05).

### Effects of PKC δ inhibition on As-induced apoptosis

To check whether there is any cross talk between PKC and MAPKs, we pre-treated the hepatocytes with rottlerin for 30 min and then studied the effects of As and taurine on JNK activation. Rottlerin has been used as a PKC*δ* inhibitor based on in vitro studies that have shown that the IC50 for PKC*δ* was 3–6 µM, PKC α,β,γ of 30–42 µM and PKC ε,η,ξ of 80–100 µM [28]. Among the protein kinases tested, only CaM-kinaseIII is suppressed by rottlerin as effectively as PKCδ [28]. Recently it has also been observed that rottlerin inhibits the Nuclear Factor *κ*B (NF-*κ*B) [29]. However, in our present study, except PKCδ no other PKC isoforms has been activated. Besides, NF*κ*B and CaM-kinaseIII were also not involved in our study. Therefore, we used rottlerin as a selective inhibitor for PKCδ. We observed that rottlerin reduced As-induced phosphorylation of PKCδ and significantly increased cell viability compared to As-induced hepatocytes (Fig. 9). Results also showed that PKCδ inhibitor blocked the As-induced JNK activation with a similar trend to the results of taurine treatment. Thus, these results suggest that taurine inhibits NaAsO_2_-induced JNK activation and apoptosis by suppressing the activation of PKCδ.

The article "Protective Role of Taurine against Arsenic-Induced Mitochondria-Dependent Hepatic Apoptosis via the Inhibition of PKCδ-JNK Pathway" was retracted in 2025. Reasons: errors in the images; duplicated images; overlap with earlier publications; original data or images not available.

**Figure 9:** Immunoblot analysis of PKCδ, JNK and cell viability in hepatocytes in response to rottlerin. Hepatyocytes were pre-treated with 10 µM rottlerin for 30 min, then treated with As (10 µM), taurine (25 mM, added 1 h prior to As treatment) for 8 h. Panel A: effect of rottlerin on Phospho and total PKCδ, Panel B: effect of rottlerin on Phospho and total JNK, Panel C: effect of rottlerin on cell viability. β actin was used as an internal control. Data represent the average ± SD of 6 separate experiments in each group. “a” indicates the significant difference between the normal control and As treated groups, “b” indicates the significant difference between the As treated and taurine treated groups. (P^a^<0.05, P^b^<0.05).

### Histological assessment

Arsenic-induced liver injury and its protection by taurine in our model are finally confirmed by the evidence of histological changes. Histological assessments of different liver segments of the normal and experimental animals have been presented in figure 10. As induced prominent hepatocytes degeneration indicated by arrows. Taurine treatment (both pre and post) showed a considerable improvement in liver morphology.

**Figure 10:** Haematoxylin and eosin stained liver section of normal, arsenic and taurine-treated rats (×10). Arrows indicate hepatocytes degeneration around the central vain in NaAsO_2_ intoxicated animals.

## Discussion

Literatures support the fact that arsenic has a direct toxic effect on cellular respiration in liver mitochondria with an evidence of oxidative stress and hepatic collagenesis in humans [30], [31], [32]. This toxic effect on cellular respiration occurs because arsenic binds to lipoic acid in the mitochondria and inhibits pyruvate dehydrogenase. The resulting uncoupling of mitochondrial oxidative phosphorylation increases hydrogen peroxide production, decreases cellular respiration and ultimately leads to hepatotoxicity and porphyrinuria. The present study also showed that exposure to sodium arsenite significantly increased ROS production, enhanced oxidative stress and induced apoptosis in hepatocytes. However, the liver conditions have been improved upon taurine treatment.

The hepatotoxic effect of As is mainly due to the depletion of GSH in the liver. In this present study, we observed several indications of oxidative stress (such as depletion of GSH, increased levels of GSSG and lipid peroxidation) in both hepatic tissues and mitochondria. Mitochondrial GSH plays an important role in maintaining mitochondria healthy and its depletion may cause oxidative injury in hepatocytes. We also found a significant increase in intracellular ROS production along with a fall in GSH generating (G6PD and GR) and ROS scavenging (antioxidant) enzymes (GST, GPx, SOD, CAT) activities in hepatic tissues. However, taurine supplementation effectively reduced these alterations in As induced hepatic pathophysiology. GSH has been considered to be an important intracellular reductant for arsenic methylation and transport [33], [34], which in turn helps the removal of arsenic from the body. Depletion of hepatic GSH facilitates accumulation of arsenic in the liver and thus causes oxidative stress. However taurine treatment significantly increased hepatic GSH level and lowered the accumulation of arsenic in hepatic tissues via increased urinary arsenic excretion. Therefore, taurine-induced increased GSH level during exposure to toxic electrophiles generated by arsenic as well as its rapid elimination/excretion from the body play an important role in decreasing oxidative stress.

The article "Protective Role of Taurine against Arsenic-Induced Mitochondria-Dependent Hepatic Apoptosis via the Inhibition of PKCδ-JNK Pathway" was retracted in 2025. Reasons: errors in the images; duplicated images; overlap with earlier publications; original data or images not available.

Apoptosis, a phenomenon of programmed cell death, is a self-destruction mechanism involved in a variety of biological events. Mitochondria have been described as the garden of cell death and play a crucial role in regulating cell death pathways [35], [36]. ROS are predominantly produced in mitochondria and play an important role in apoptosis. The central executers of the apoptotic pathways are Bcl-2 family proteins and caspases (cysteinyl aspartic acid-specific proteases). Bcl-2 family members regulate apoptosis by modulating the release of cytochrome c from mitochondria to cytosol. In the cytosol, Apaf1, procaspase-9 and released cytochrome c from the mitochondria interact to form the apoptosome that drives the activation of caspase-3. To confirm As-induced mitochondria-dependent apoptosis, we determined the mitochondrial membrane potential, intracellular ATP level as well as expressions of Bcl-2 family and BH-3 only proteins, cytochrome c, caspase 3, caspase 9, Apaf1 and PARP in arsenic-induced hepatic pathophysiology and observed that As significantly up-regulated pro-apoptotic (Bad, Bax, Bim) and down-regulated anti-apoptotic (Bcl-2, Bcl-xL) proteins, reduced mitochondrial membrane potential and intracellular ATP level, increased cytochrome c release and protein level of Apaf-1 in the cytosol. Reduction of the mitochondrial membrane potential and activation of caspases (caspase 3 and caspase 9) subsequently modulated PARP cleavage from its full-length form (116 kDa) to the cleaved form (84 kDa). In liver, arsenic also markedly enhances cellular Bax and reduces Bcl-2 mRNA levels and therefore probably regulates Bax and Bcl-2 expression by both transcriptional and post-transcriptional levels. Taurine treatment, however, effectively inhibited all these As-induced pro-apoptotic events.

The article "Protective Role of Taurine against Arsenic-Induced Mitochondria-Dependent Hepatic Apoptosis via the Inhibition of PKCδ-JNK Pathway" was retracted in 2025. Reasons: errors in the images; duplicated images; overlap with earlier publications; original data or images not available.

MAPKs comprise a family of serine/threonine phosphorylating proteins that mediate a variety of signal transduction pathways [37], [38]. Among the MAPKs, the c-Jun NH2-terminal kinases (JNKs) and p38 result in stress responses, growth arrest, and/or apoptosis. Therefore, in order to investigate the underlying mechanisms of apoptosis in As intoxicated liver (and hepatocytes) and the beneficial role of taurine in this hepatic pathophysiology, we investigated the changes in the levels of ERK1/2, p38 and JNK by immunoblot analyses. We observed a marked increase in protein content of phosphorylated p38 MAPK and JNK in As-intoxicated liver and hepatocytes. A marginal increment of pERKs was also noted in both the liver and hepatocytes. We also observed that, hepatocytes treated with JNK inhibitor SP600125, suppressed the As-induced caspase 3 activation, cell viability reduction and ROS production. However, a p38-MAPK specific inhibitor, SB203580, had no effect on cell viability and caspase 3 activation on hepatocytes exposed to As. The present study also showed that taurine treatment prevented As-induced activation of Bim-EL in liver and hepatocytes. Therefore, we can conclude that JNK may induce hepatocyte apoptosis via a Bim-mediated, Bax-dependent mitochondrial pathway of cell death. These observations are in consistent with the data of other models where JNK-dependent Bim induction as well as phosphorylation with downstream activation of Bax-mediated apoptosis have been reported [39], [40].

Protein kinase C (PKC) is a family of enzymes that are involved in controlling the function of other proteins through the phosphorylation of hydroxyl groups of serine and threonine amino acid residues on those proteins. PKC family consists of at least 12 members and can be classified into three groups based on their biochemical properties and sequence homologies, e.g. conventional PKC isoforms (cPKC-α,-βI,-βII,-γ), novel PKC isoforms (nPKC –δ,–ε,–μ,–η,–θ) and atypical PKC isoforms (aPKC-λ,–ι,–ξ). The different PKC isoforms might have specific roles in signal transduction. In our study, western blot analyses revealed that NaAsO_2_ intoxication significantly increased the expression of PKCδ both in liver tissues and hepatocytes with out changing the expression of other two major isoforms, PKCα and PKCξ. However, treatment with taurine markedly suppressed this As-induced phosphorylation of PKCδ. Furthermore, the decreased JNK activity by the specific inhibitor of PKCδ, rottlerin, strongly suggests the involvement of PKCδ in As-induced JNK activation. Further studies will clarify the exact activation mechanisms of PKCδ in response to ROS. However, one possible explanation is the production of intracellular H_2_O_2_ due to NaAsO_2_ intoxication, which subsequently activates PKCδ [41], [42]. As taurine treatment reduced the hepatic H_2_O_2_ production, As-induced PKCδ activation was also suppressed.

The article "Protective Role of Taurine against Arsenic-Induced Mitochondria-Dependent Hepatic Apoptosis via the Inhibition of PKCδ-JNK Pathway" was retracted in 2025. Reasons: errors in the images; duplicated images; overlap with earlier publications; original data or images not available.

As-induced liver injury in this model is also supported by the histological changes and the increased arsenic content in the liver tissue of the intoxicated animals. However, taurine could effectively prevent the As-induced alterations of hepatic morphology and increased the excretion of As from the liver tissues.

In summary, our study demonstrates a pivotal role of mitochondria in hepatocytes apoptosis. Reactive oxygen species generated during NaAsO_2_ exposure, induce PKCδ activation, which subsequently activates JNK and helps the progression of apoptosis. Taurine treatment, on the other hand, attenuates As-induced oxidative stress in the liver and thus prevents hepatic apoptosis. This anti-apoptotic effect of taurine is mediated by blocking the activation of PKCδ and JNK, generation and accumulation of ROS and elimination/excretion of As from the body. Taken together, our findings outline a mechanistic understanding of how taurine protects liver from As-induced toxicity (Fig. 11). In conclusion, present experimental findings point out the importance of the chronology for the treatment outcome and provided the protection that taurine could afford against arsenic-induced hepatic dysfunction by its antioxidant potential as well as other pathways involved in apoptotic cell death.

**Figure 11:** Schematic diagram of the NaAsO_2_ induced hepatotoxicity and its prevention by taurine.

## Materials and Methods

### Chemicals

Taurine (2-aminoethane sulfonic acid), anti Caspase-3, anti Cleaved Caspase-3, anti PARP, anti Apaf-1 antibodies were purchased from Sigma-Aldrich Chemical Company (St. Louis, USA). Anti BAD and anti Bcl-2 were purchased from Santa Cruz Biotechnology (Santa Cruz, CA). Sodium arsenite (NaAsO_2_) was bought from Sisco Research Laboratory (Mumbai, India).

### Animals

Swiss albino adult male rats weighing approximately 200–250 g and albino mice of Swiss strain, weighing between 20–25 g were were purchased from M/S Gosh Enterprises, Kolkota, India. Animals were acclimatized under laboratory condition for two weeks prior to the experiments. All the experiments with animals were carried out according to the approval and guidelines of the Bose Institute animal ethical committee (the permit number is: 95/99/CPCSEA).

### Determination of dose for As induced hepatic dysfunctions *in vivo*

To establish the dose of As necessary for hepatic damage, rats were randomly allocated into seven groups each consisting of six rats and they were treated as follows. First group served as normal control (received only water as vehicle). Remaining six groups were treated with six different doses of NaAsO_2_ orally (0.5 mg, 1 mg, 1.5 mg, 2 mg, 2.5 mg and 3 mg/kg body weight in distilled water for 6 months).

The article "Protective Role of Taurine against Arsenic-Induced Mitochondria-Dependent Hepatic Apoptosis via the Inhibition of PKCδ-JNK Pathway" was retracted in 2025. Reasons: errors in the images; duplicated images; overlap with earlier publications; original data or images not available.

Twenty-four hours after the final dose of NaAsO_2_ intoxication, all rats were sacrificed and ALP levels were measured using serum of all experimental rats.

### Determination of dose and time dependent activity of taurine by ALP assay

For this study, rats were randomly distributed into eight groups each consisting of six animals. First two groups were served as normal control (received only water as vehicle) and toxin control (received 2 mg/kg body weight for 6 months, orally) respectively. Remaining six groups of animals were treated with six different doses of taurine (10mg, 20mg, 30mg, 40 mg, 50mg and 60mg/kg body weight for 2 weeks, orally in distilled water) followed by NaAsO_2_ intoxication (received 2 mg/kg body weight for 6 months, orally).

To determine the time dependent effects of taurine for pre-treatment in NaAsO_2_-dependent hepatic disorder, rats were divided into eight groups each consisting of six animals. First two groups were served as normal control (received only water as vehicle) and toxin control (received 2 mg/kg body weight for 6 months, orally) respectively. Other seven groups of animals were treated with taurine orally at a dose of 50 mg/kg body weight, once daily for 0.5,1, 1.5, 2, 2.5 and 3 weeks prior to NaAsO_2_ intoxication (received NaAsO_2_ at a dose 2 mg/kg body weight for 6 months, orally).

Similarly, to determine the time dependent effects of taurine for post-treatment studies in NaAsO_2_-dependent hepatic disorder, rats were divided into eight groups each consisting of six animals. First three groups were served as normal control (received only water as vehicle), toxin control (received 2 mg/kg body weight for 6 months, orally) and recovery (received 2 mg/kg body weight for 6 months, orally and received normal diet for next 2 weeks) respectively. Other five groups of animals were treated with taurine orally at a dose of 50 mg/kg body weight, once daily for 0.5, 1, 2, 2.5 and 3 weeks after NaAsO_2_ administration (received 2 mg/kg body weight for 6 months, orally).

At selected times after NaAsO_2_ and taurine treatment, all rats were sacrificed. ALP levels were measured using serum of all experimental rats.

### *In vivo* experimental set-up

The animals were divided into five groups, consisted of six rats in each and they were treated for 14 weeks as follows.

The article "Protective Role of Taurine against Arsenic-Induced Mitochondria-Dependent Hepatic Apoptosis via the Inhibition of PKCδ-JNK Pathway" was retracted in 2025. Reasons: errors in the images; duplicated images; overlap with earlier publications; original data or images not available.

Group 1: “Normal control”: animals received only water as vehicle.

Group 2: “Toxin control (As)”: animals received 2 mg/kg body weight once daily for 6 months, orally.

Group 3: “Taurine pre-treated group (TAU+As)”: animals were treated with taurine (orally, 50 mg/kg body weight in distilled water, once daily) for 2 weeks followed by NaAsO_2_ intoxication for 6 months.

Group 4: “Taurine post-treated group (As+TAU)”: received NaAsO_2_ for 6 months followed by taurine administration at a dose of 50 mg/kg body weight in distilled water once daily for 2 weeks.

Group 5: “Taurine alone treated group (TAU)”: animals were treated with taurine (orally, 50 mg/kg body weight in distilled water, once daily) for 2 weeks followed by no treatment for next 6 months.

The animals were sacrificed under light ether anesthesia and livers were collected.

### Determination of liver weight to body weight ratio

After sacrification, the livers from experimental animals were quickly excised and weighed. Then the ratio of liver weight to body weight was measured for each.

### Hepatic and urinary arsenic estimation

The arsenic contents in liver tissues and urinary assenic level of all experimental animals were analyzed following the method of Das et al [43] using hydride generation system in Atomic Absorption Spectrophotometer (Perkin Elmer Model No. 3100).

### Assessment of serum specific markers related to hepatic dysfunction

For assessment of serum specific markers (ALT and ALP levels) related to hepatic dysfunction, blood samples were collected by puncturing rat hearts of all experimental animals, kept overnight for clotting and then centrifuged at 3,000 g for 10 minutes. ALT and ALP levels in the serum were measured by using standard kits according to the method of Rietman and Frankel [44] and Kind and King [45] respectively.

### Preparation of liver homogenate

Liver samples were homogenized using glass homogenizer in 100 mM potassium phosphate buffer containing 1 mM EDTA, pH 7.4 supplemented with protease and phosphatase inhibitors and centrifuged at 12,000 g for 30 minutes at 4°C. The supernatant was collected and used for the experiments.

### Determination of protein content

The protein content of the experimental samples was measured by the method of Bradford [46] using crystalline BSA as standard.

### Assay of cellular metabolites

Reduced glutathione (GSH) level was measured following the method of Ellman [47] by using DTNB (Ellman's reagent) as the key reagent. Oxidized glutathione GSSG contents in the hepatic tissues of the experimental and normal animals were determined following the method of Hissin and Hilf [48].

The article "Protective Role of Taurine against Arsenic-Induced Mitochondria-Dependent Hepatic Apoptosis via the Inhibition of PKCδ-JNK Pathway" was retracted in 2025. Reasons: errors in the images; duplicated images; overlap with earlier publications; original data or images not available.

### Measurement of lipid peroxidation

The lipid peroxidation in terms of malondialdehyde (MDA) formation was measured according to the method of Esterbauer and Cheeseman [49].

### Estimation of hepatic H_2_O_2_ level

The hydrogen peroxide level in liver tissue was determined using a slightly modified ferrous thiocyanate method of Chen et al [50].

### Assay of antioxidant enzymes

The activities of antioxidant enzymes, SOD, CAT, GST, GR, GPx and G6PD have been measured in liver homogenates of all experimental animals.

SOD activity has been measured by following the method originally developed by Nishikimi et al [51] and then modified by Kakkar et al [52].

CAT activity was determined by following the decomposition of H_2_O_2_ at 240 nm for 10 minutes and it was monitored spectrophotometrically according to the method of Bonaventura et al [53].

GST activity was assayed based on the conjugation reaction with glutathione in the first step of mercapturic acid synthesis Habig et al [54].

GR activity was determined according to the method of Smith et al [55]. The increase in absorbance at 412 nm was monitored spectrophotometrically for 3 minutes at 24°C.

GPx activity was measured by following the method of Flohe and Gunzler [56] using H_2_O_2_ and NADPH as substrates.

G6PD activity was determined as described by Lee [57].

### Detection of cell death pathway by flowcytometry, DNA fragmentation assay and DAPI staining

Hepatocytes were isolated from arsenic and taurine treated rat liver by perfusion technique with collagenase type I at 37°C [58]. Cells were washed with PBS, centrifuged at 800 g for 6 min, resuspended in ice-cold 70% ethanol/PBS, centrifuged at 800 g for a further 6 min, and resuspended in PBS. Cells were then incubated with propidium iodide (PI) and FITC-labelled Annexin V for 30 min at 37°C. Excess PI and Annexin V were then washed off; cells were fixed and then stained cells were analyzed by flow cytometry using FACS Calibur (Becton Dickinson, Mountain View, CA) equipped with 488 nm argon laser light source; 515 nm band pass filter for FITC-fluorescence and 623 nm band pass filter for PI-fluorescence using CellQuest software.

The DNA fragmentation has also been assayed by electrophoresing genomic DNA samples, isolated from normal as well as experimental rat liver as above, on agarose/EtBr gel by the procedure described by Sellins and Cohen [59].

To detect morphological evidence of apoptosis, cell nuclei were visualized following DNA staining with the fluorescent dye DAPI [60]. Hepatocytes isolated from NaAsO_2_ and taurine treated rats as above were incubated for 10 min with DAPI (1 µg/ml) and examined using fluorescent microscopy (Microphot FX; Nikon, Tokyo).

The article "Protective Role of Taurine against Arsenic-Induced Mitochondria-Dependent Hepatic Apoptosis via the Inhibition of PKCδ-JNK Pathway" was retracted in 2025. Reasons: errors in the images; duplicated images; overlap with earlier publications; original data or images not available.

### Hepatocyte isolation and *in vitro* experimental protocol

Hepatocytes were isolated from rat liver following the method of [58] with some modifications. Hepatocytes were then treated with taurine (25mM), NaAsO_2_ (10 µM) and taurine coupled (1h before) with NaAsO_2_ and incubated at 37°C for 8 hours for further molecular and biochemical analyses.

### Cell viability assessment

About 2×10^6^ hepatocytes were incubated with As either alone or after taurine administration following the method of Madesh and Balasubramanian [61]. The tetrazolium salt MTT can be used to measure the metabolic activity of viable cells. Tetrazolium salts are reduced to formazan by mitochondrial succinate dehydrogenase, an enzyme which is only active in cells with an intact metabolism and respiratory chain. The formazan is quantified photometrically and correlates with the number of viable cells.

### Measurement of intracellular ROS production

Briefly, hepatocytes were incubated with DCF-DA (10 mM) for 1 h at 37°C in the dark. After treatment, the cells were immediately washed and resuspended in PBS. Intracellular ROS production was detected using the fluorescent intensity of the oxidant sensitive probe 2,7dichlorodihydrofluorescein diacetate (H_2_DCFDA) in a fluorescence microscope.

### Determination of mitochondrial membrane potential (Δψ_m_)

After experimental treatment and following the method of Hodarnau et al. [62], fresh mitochondria were isolated from the liver tissue. Mitochondrial membrane potential (Δψ_m_) was estimated [63] on the basis of cell retention of the fluorescent cationic probe rhodamine 123. The results are expressed as percentage of the fluorescence values for control (untreated).

### Intracellular ATP determination

Hepatocytes that were left untreated or treated with As alone or pretreated with taurine were used for analysis of intracellular ATP as described by Kalbheim and Koch [64].

### Immunoblotting

For immunoblotting, samples containing 50 µg proteins were subjected to 10% SDS-PAGE and transferred to a nitrocellulose membrane. Membranes were blocked at room temperature for 2 h in blocking buffer containing 5% non-fat dry milk to prevent non specific binding and then incubated with anti Bim-EL (1∶1000 dilution), anti BAD (1∶1000 dilution), anti Bcl-2 (1∶1000 dilution), anti cytochrome c (1∶1000 dilution), anti cleaved caspase9 (1∶1000 dilution), anti-cleaved caspase3 (1∶250 dilution), Apaf-1(1∶1000 dilution), anti-PARP (1∶1000 dilution), anti p-38 (1∶1000 dilution), anti ERK1/2 (1∶1000 dilution), anti p-JNK (1∶1000 dilution), PKCδ (1∶1000 dilution), PKCα (1∶1000 dilution) and PKCξ (1∶1000 dilution), primary antibodies at 4°C overnight. The membranes were washed in TBST (50 mmol/L Tris-HCl, pH 7.6, 150 mmol/L NaCl, 0.1% Tween 20) for 30 min and incubated with appropriate HRP conjugated secondary antibody (1∶2000 dilution) for 2 h at room temperature and developed by the HRP substrate 3,3′-diaminobenzidine tetrahydrochloride (DAB) system (Bangalore, India).

The article "Protective Role of Taurine against Arsenic-Induced Mitochondria-Dependent Hepatic Apoptosis via the Inhibition of PKCδ-JNK Pathway" was retracted in 2025. Reasons: errors in the images; duplicated images; overlap with earlier publications; original data or images not available.

### RNA extraction and RT-PCR

RNA was extracted from liver that were left untreated or treated with As alone or treated with taurine using the Trizol method. One microgram of RNA was converted to cDNA using superscript reverse transcriptase. Thermal cycling was performed as follows: 95°C for 105 s (initial denaturation) followed by the set of cycles: 95°C for15 s (denaturation), 55°C for 30 s (primer annealing), 72°C for 30 s (primer extension). After 25 cycles the time of DNA extension was 7 min at 72°C. The PCR amplification products were then cooled at 4°C. The PCR amplified products were then subjected to electrophoresis on 1.5% agarose gels. The product size and annealing temperature of the primers used were given in table 5.

**Table 5:** Primers used for Bax, Bcl-2 and β-actin genes.

Gene	Oligonucleotides used for real-time polymerase chain reaction (PCR) primer sequence 5′ to 3′	Annealing temperature (°C)	Product Size(bp)
Bax	Fp: 5′-GGTTGCCCTCTTCTACTTT-3′Rp: 5′-AGCCACCCTGGTCTTG-3′	55	143bp
Bcl-2	Fp: 5′-ACTTTGCAGAGATGTCCAGT-3′Rp: 5′-CGGTTCAGGTACTCAGCAT-3′	55	217 bp
β-actin	Fp: 5′- CGTTGACATCCGTAAAGAC-3′Rp: 5′--TAGGAGCCAGGGCAGTA-3′	55	110bp

### Histological studies

Livers from the normal and experimental rats were fixed in 10% buffered formalin and were processed for paraffin sectioning. Sections of about 5 µm thickness were stained with haematoxylin and eosin to evaluate under light microscope.

### Statistical Analysis

All the values are expressed as mean ± S.D. (n = 6). Significant differences between the groups were determined with SPSS 10.0 software (SPSS Inc., Chicago, IL, USA) for Windows using one-way analysis of variance (ANOVA) and the group means were compared by Duncan's Multiple Range Test (DMRT). A difference was considered significant at the p<0.05 level.
